The article "Brain tumor recognition by an optimized deep network utilizing ammended grasshopper optimization" was published in 2024. Journal: Heliyon.

# Brain tumor recognition by an optimized deep network utilizing ammended grasshopper optimization

**DOI:** 10.1016/j.heliyon.2024.e28062

**Published:** 2024-03-24

**Authors:** Jing Zhu, Chuang Gu, Li Wei, Hanjuan Li, Rui Jiang, Fatima Rashid Sheykhahmad

**Affiliations:** a Department of Radiology, The General Hospital of Western Theater Command, Chengdu, 610083, Sichuan, China; b Department of Radiology. The General Hospital of The General Hospital of The 964th Hospital, Changchun, 130000, Jilin, China; c Nursing Department. The General Hospital of The 964th Hospital, Changchun, 130000, Jilin, China; d Ardabil Branch, Islamic Azad University, Ardabil, Iran; e College of Technical Engineering, The Islamic University, Najaf, Iraq

**Keywords:** Brain tumor, Diagnosis, AlexnNet, Extreme learning machine, Convolutional neural network, Ammended grasshopper optimization algorithm

## Abstract

Brain tumors are abnormal cell masses that can get originated in the brain spread from other organs. They can be categorized as either malignant (cancerous) or benign (noncancerous), and their growth rates and locations can impact the functioning of the nerve system. The timely detection of brain tumors is crucial for effective treatment and prognosis. In this study, a new approach has been proposed for diagnosing brain tumors using deep learning and a meta-heuristic algorithm. The method involves three main steps: (1) extracting features from brain MRI images using AlexNet, (2) reducing the complexity of AlexNet by employing an Extreme Learning Machine (ELM) network as a classification layer, and (3) fine-tuning the parameters of the ELM network using an Amended Grasshopper Optimization Algorithm (AGOA). The performance of the method has been evaluated on a publicly available dataset consisting of 20 patients with newly diagnosed glioblastoma that is compared with several state-of-the-art techniques. Experimental results demonstrate that the method achieves the highest accuracy, precision, specificity, F1-score, sensitivity, and MCC with values of 0.96, 0.94, 0.96, 0.96, 0.94, and 0.90, respectively. Furthermore, the robustness and stability of the method have been illustrated when subjected to different levels of noise and image resolutions. The proposed approach offers a rapid, accurate, and dependable diagnosis of brain tumors and holds potential for application in other medical image analysis tasks.

## 1 Introduction

A set of abnormal cells cause a brain tumor in the brain. The brain is surrounded by skull, which is very hard. With any growth in this space, some problems appear. Malignant or benign are two kinds of tumors in brain. When cancerous or non-cancerous tumors grow, intracranial pressure increases that can cause brain hurt and can be dangerous. The rate of tumor growth in brain is very different. The functioning of the system of nerves has been influenced by the proportion of progress and the position of the brain tumor. Primary or secondary are the classification of these tumors [1]. The source of initial brain tumor has been considered to be from brain [2]. Myriad cases of these tumors are non-cancerous. Metastatic brain tumors, which are second brain tumors, ger originated from other organs, including the breast or lungs to the brain.

Among different bio-medical researches, the detection of brain tumors is, perhaps, a key challenge. As a result, the early detection has been found to be essential for treatments and increasing survival [3]. The vital parameters of detection are patient's medical history, findings of laboratory, physical examination, and mainly imaging [4]. Most of the methods of diagnostic imaging are applied to recognize any unusual alterations in tissues and organs, which are CT (Computed Tomography) scans and MRI (Magnetic Resonance Imaging). However, as previously mentioned, the imaging is a most significant part of the brain tumor detection that in some cases, experts do wrong diagnosis which can be so harmful for the patient. On the other hand, literature shows that computer vision technology, without human intervention, provides more accurate results in different cases [4]. Therefore, this can be an efficient technique to help the experts increase precision of their diagnosis. Different studies are done within the present category. To exemplify, Gurbină et al. [5] focused on the intricate nature of the brain and its billions of cells. Their main objective was to address the issue of cerebral tumors, which occurred when cells divide uncontrollably and formed abnormal cell groups in or around the brain. These abnormal cell groups can disrupt normal activity of brain and cause harm to healthy cells. The tumors are classified as benign or low-grade and malignant or high-grade. The proposed methodology aimed to differentiate between normal brains and those with the presence of tumors, whether benign or malignant. To achieve this, the researchers utilized brain Magnetic Resonance Imaging (MRI) and employed various wavelet transforms and Support Vector Machines (SVM) for the detection and classification of different types of brain tumors, such as metastatic bronchogenic carcinoma tumors, glioblastoma, and sarcoma. The accurate and automated classification of MRI brain images is crucial for medical analysis and interpretation. However, it is important to acknowledge the limitations of this study. Firstly, the effectiveness of the proposed methodology might be influenced by factors, such as the size and location of the tumors as well as individual variations among patients. Additionally, the generalizability of the findings might be limited due to the specific types of tumors that were studied. It would be advantageous to explore a wider range of tumor types to enhance the applicability of the methodology. Furthermore, the study relied on a specific combination of wavelet transforms and SVMs, and alternative algorithms might yield different results. Lastly, the accuracy of the automated classification system should be validated through extensive testing and comparison with expert human interpretations.

Sathish et al. [6] focused on the classification of tumor regions in MRI brain imaging. They proposed a Radial Basis Neural Network (RBNN) based on an exponential cuckoo search algorithm for the automatic classification of brain tumors. The process involved using fuzzy c-means clustering for tumor region segmentation and extracting features from both tumor and non-tumor regions to generate a feature vector. These features were, then, used by the RBNN classifier, which required optimal cluster centers determined by the newly proposed exponential cuckoo search algorithm. The classifier successfully classified tumor and non-tumor images and determined the severity of the tumor. The proposed system achieved a high accuracy of 89% for the classification of MRI brain images. However, there are limitations to consider. Firstly, the effectiveness of the proposed method may vary depending on the size, location, and characteristics of the tumors, as well as individual patient variations. Additionally, the study only focused on brain tumors and did not consider other types of tumors that could be present in the MRI images. It would be valuable to explore the generalizability of the system to a broader range of tumors. Moreover, the proposed algorithm relied on specific clustering and classification techniques, and alternative methods might yield different results. Finally, the evaluation metrics used in the study should be validated through further testing and comparison with expert interpretations to ensure their reliability and applicability in real-world clinical settings.

Kumar et al. [7] designed a combined DNN model and PDIM (Pyramid Design of Inception Module) for image segmentation of brain by MRI. In the DNN model, convolution filters of various sizes caused problems in updating the weight and overfitting due to the effect on the abstract properties of the input variables. To address these shortcomings, a conventional Inception Module (IM) module with a broader and deeper architectural design was used. The finding presented that the designed model reached 99% of precision, 98% of sensitivity, and 100% of specificity. The results showed that the operation of a system was designed to help physicians precisely classify the brain tumor.

Khairandish et al. [8] introduced combined CNN-SVM methods for segmentation of brain images on MRI to diagnose brain cancer. One of the methods of identifying tumors in brain is MRI (Magnetic Resonance Imaging). In this research, combined CNN-SVM methods were used to detect abnormal cells in the brain. The results of comparing the introduced model with Rough Extreme Learning Machine (RELM), Deep Neural Network (DNN), Deep CNN (DCNN) and automatic Discrete Wave Encoder (DWA), CNN, K-Nearest Neighbors (KNN), and CNN-SVM were evaluated. The accuracy of each of these models was 94.233%, 95%, 96%, 97.5%, 98.4959%, respectively. Estimations showed that the CNN-SVM model was able to identify abnormal cells in the brain more accurately.

Cristin et al. [9] detected brain cancer by MRI images applying a fractional-Chicken Swarm Optimizer. Early detection of brain cancer could lead to earlier treatment of the disease and prevent an increase in mortality of the disease. The innovation of the study was an optimized deep recurrent neural network based on Fractional-Chicken Swarm Optimization Algorithm to identify cancer cells of the brain. The results of evaluation metrics showed that the precision, specificity, and sensitivity of this model were 93.35%, 96%, and 95%, respectively. The estimated values showed that the proposed model was satisfactory in identifying cancer cells in the brain.

Irmak et al. [10] applied a Hybrid DCNN based on a Fully Optimized Framework to detect abnormal cells of the brain. Three various CNN techniques were used for three different categorization tasks in this paper. All CNN models were optimized using the network's fully optimized framework. The first designed model was able to identify brain cells with 99.33% precision. The second CNN model was able to identify abnormal brain cells with 92.66% precision. The other technique was able to identify brain tumors with 98.14% precision. CNN's introduced models were compared to other techniques like GoogleNet ResNet-50, VGG-16, Inceptionv3, and AlexNet. The comparison achievements indicated the good operation of these models in the identification and categorization of cancerous tumor. Therefore, this model could have acceptable effectiveness in the field of medicine and radiology.

Sultan et al. [11] suggested a categorization technique on images of brain tumor using Deep Neural Network to identify tumors for earlier treatment. In this study, a newer technique was proposed to identify cancerous tumors in the brain. This method was the data-driven method that was called Convolutional Neural Network (CNN). This model could be used to segment MRI images to detect abnormal cells of the brain. The achievements indicated that this technique revealed the precision of 96.13% and 98.7% for the two case studies. Therefore, they presented CNN model with the best performance for detecting cancer cells in the brain.

These methods can be used also in different applications [12]. According to the literature, however, various techniques have been established for better detection of brain tumor, there is still gap in providing more accurate methods. By analyzing the literature above, it can also concluded that most of the newest approaches are based on the metaheuristic-based algorithms that showed high accuracy in the brain tumor diagnosis.

In this study, a new and efficient method has been introduced for diagnosing brain tumors. The method utilizes a metaheuristic-based deep network, which is a novel approach. The method combines an AlexNet for extracting features with Extreme Learning Machine (ELM) network for classification,.

Both AlexNet and ELM are widely recognized as efficient methods for diagnosing brain tumors using MRI images. AlexNet has the ability to automatically extract features from images, eliminating the need for manual feature engineering. On the other hand, ELM is an extreme learning machine that can classify data with a single hidden layer and random weights, without requiring iterative training.

Utilizing AlexNet and ELM for brain tumor diagnosis offers several advantages. Firstly, AlexNet excels at capturing intricate and advanced features from brain MRI images, thereby enhancing the accuracy and robustness of the diagnosis. Secondly, ELM simplifies the complexity and computational burden of AlexNet by replacing the last few layers with a straightforward and rapid classifier.

Moreover, ELM addresses common issues encountered in traditional neural networks, such as overfitting, local minima, and gradient vanishing. By avoiding these problems, ELM ensures more reliable and stable results in the diagnostic process.

To further enhance the performance of AlexNet and ELM, a modified meta-heuristic algorithm, called amended grasshopper optimization algorithm, is employed to aid in fine-tuning the parameters and optimizing the overall performance of both techniques.

## 2 Materials and methods

For designing an efficient method to diagnose the brain tumor, an optimized system is utilized on the basis of deep learning. All of the simulations have been conducted within the MATLAB R2019b, and their outcomes have been authenticated through being applied to a database.

### 2.1 Dataset

The dataset utilized in this paper is “Brain-Tumor-Progression” [13]. This dataset comprises Magnetic Resonance Imaging (MRI) data obtained from 20 patients who have recently been diagnosed with glioblastoma, an aggressive form of brain tumor. The data were obtained from The Cancer Imaging Archive (TCIA), a publicly accessible repository of cancer-related imaging data. The primary objective of this dataset is to assess the effectiveness of deep learning algorithms in predicting tumor progression. Each patient's data include two MRI scans: one taken within 90 days after completing standard Chemo-Radiation Therapy (CRT) and another at the time of tumor progression, as determined by clinical and/or imaging. The MRI scans encompass various modalities, such as T1-weighted (T1w), T2-weighted (T2w), Fluid-Attenuated Inversion Recovery (FLAIR), Apparent Diffusion Coefficient (ADC), and perfusion images. The perfusion images were acquired using Dynamic Susceptibility Contrast (DSC) imaging with a contrast agent preload. Additionally, the dataset provides binary tumor masks that identify regions of abnormal tissue on the T1w images. All image series in the dataset are co-registered with the T1w images featuring contrast (T1+C) enhancement and are stored in DICOM format. The dataset has a total size of 3.2 GB and encompasses 383 image series and 8798 images.

Having access to the dataset requires a restricted license agreement to protect the privacy of the participants. This dataset can be downloaded from the following link: https://doi.org/10.7937/K9/TCIA.2018.15quzvnb.

Here, 7038 images (about 80%) has been used for training the network, and 1760 number of images (about 20%) has been used for testing the network. Fig. (1) shows some examples of the Brain-Tumor-Progression dataset.

**Fig. 1:** Some examples of the Brain-Tumor-Progression dataset.

### 2.2 AlexNet

Alexnet is a type of CNN that gained the prize of the Imagenet challenge in 2012 [1]. This network was desiged by Krizhevsky et al. [14].

There are 8 deep layers and 5 layers in the Alexnet. The network uses max pooling technique that is followed by three fully related layers. The ReLU (Rectified Linear Unit) is the function of activation such that f(x) = max(x,0) [10]. The reason for using ReLU in this network is to speed up the training process for about 6 times. The method of scale reduction in this study is Max pooling. The network also utilized dropout layers to prevent from overfitting [15]. The input size for the AlexNet is 227×227. Therefore, all input images in this study were converted to this size before training and validation.

The first layer of convolution is a 96-filter with 11×11. The padding for this layer has 2 pixels and the stride has 4 pixels. Although, the next convolutional layers' stride and padding are set to 1 pixel. 256 filters of the size have been have been used to the second convolutional layer [16]. Then, with the same size of 3 × 3, 384 filters are used for the third, 384 filters have been used for fourth, and 256 filters have been used for fifth convolutional layers. Here, to improve the consistency of the proposed AlexNet in diagnosing the brain tumor, Batch Normalization (BN) procedure has been utilized. This approach also helps enhance the network's speed. Due to different intensity and the large number of the images, the network's complexity is too much which reduces its speed a lot [3]. Fig. (2) shows the architecture of AlexNet.

**Fig. 2:** Architectures of AlexNet.

By training the convolutional neural network using minibatch methodology, a normalization transform has been employed by the layer of activations for remembrancing the variances and constant means [17]. Therefore, by random assessment of the variables set, ($z_{i}:i=1,2,\ldots ,n)$ and assuming mb as mini-batch values, the mean (${\bar{Z}}_{mb}$) and the standard deviation ($S_{mb}^{2}$) values have been accomplished through the subsequent formulation [equations (1), (2)]:

(1) $${\bar{Z}}_{mb}=\frac{1}{N}\sum_{j=1}^{N}z_{i}$$

(2) $$S_{mb}^{2}=\frac{1}{N}\sum_{j=1}^{N}{\left(z_{i}-{mean}_{S}\right)}^{2}$$

where, ${\bar{Z}}_{mb}$ describes the mean values, $S_{mb}^{2}$ defines the standard deviation values, $mb=\left[z_{1},z_{2},\ldots ,z_{n}\right]$ represents the mini-batch values, and the normalized value ($\hat{z_{i}}$) has been modeled by equation (3):

(3) $$\hat{z_{i}}=\frac{z_{i}-{\bar{Z}}_{mb}}{\sqrt{S_{mb}^{2}+\varepsilon }}$$

where, ε defines a too small value to escape from steadiness.

Because the learning target is not to normalize the activations, the succeeding transformation has been employed [equation (4)]:

(4) $$y_{i}=a+b\times {\hat{z}}_{i}$$

where, a and b represent two tunable parameters.

By using the batch normalization, the training speed of the network has increased.

### 2.3 Extreme learning machine (ELM)

Here, AlexNet is used for the diagnois of the brain tumor. However, due to the dependence of this network on the earlier entirely linked layers, providing a modification for better results is mandatory. This is established by combining this network with ELM. This is a feedforward neural network. This has been, first, introduced by G. Huang [18]. The main advantage of the Extreme Learning Machine is that it does not need gradient-based backpropagation. Instead, it uses another method, called “Moore-Penrose generalized inverse” for quantification of the network's weights.

An Extreme Learning Machine can be considered as a fast way to train Single hidden Layer Feedforward Network (SLFN). SLFNs contain 3 layers of neurons which include 1 layer with non-linear neurons within the concealed layer. The input layer delivers features of the data, while the output layer with linear architecture does not have transformation function. Fig. (3) displays a general ELM model.

**Fig. 3:** A general ELM model.

The weights of input (W), output weights (β), and the biases (b) in this network are set randomly with no adjustrment which makes it so faster than the other techniques in evaluating the linear output layer. This study uses ELM alongside the AlexNet to provide a more efficient network for diagnosing the brain tumors. The ELM also helps AlexNet to use much less number of iterations for training.

By considering x and O as inputs and outputs of the network, a training set M has been signified subsequently [equation (5)]:

(5) $$M=\left[\left(x_{1},t_{1}\right),\left(x_{2},t_{2}\right),\ldots ,\left(x_{n},t_{n}\right)\right]$$

where, $x_{i}$ and $t_{i}$ describe, in turn, the vector of input and the label.

The matrix of output for concealed layer H is accomplished as follows [equation (6)]:

(6) $$H=\sum_{l=1}^{M}f_{i}\times \left(w_{i}x_{i}+b_{i}\right)$$

where, l=1,2,…,L*,* f(.) specifies the function of activation for the concealed layer, and M defines the quantity of concealed nodes. The aim is to provide the output of the network, as sample labels are expressed in the following way [equation (7)]:

(7) Hρ=T

where, $T=\left[t_{1},t_{2},\ldots ,t_{L}\right]$, and ρ is achieved by equation (8):

(8) $$\rho =H^{†}T$$

where, T specifies the sample labels that are the desired output of the network, H is the matrix of output considering concealed layer, and † signifies the pseudo-inverse operator.

As was previously mentioned, the model of ELM is employed to replace the previous layers to reduce the system's complexity during the diagnosis process. As mentioned before, ELM uses random values for all weights and biases. Here, for providing optimal results of the current research, the biases and weights have been chosen by a recent enhanced design of Grasshopper Optimizer.

## 3 Amended grasshopper optimization algorithm

### 3.1 Introduction of grasshopper optimizer

One of the main and vital issues in technology and science is optimization; therefore, various algorithms with metaheuristic approaches have been introduced in this regard [19]. Recetly, lots of metaheuristic algorithms have been presented for the engineering applications [20]. Also, there are some modifications of these types of algorithms to improve their efficiency in different terms [[21], [22], [23]]. The Grasshopper Optimization Algorithm (GOA) is a new metaheuristic. The algorithm is simple and has only one setting parameter: the grasshoppers are insects that live in groups [24]. Their group manner of living can be discovered in adult grasshoppers and baby grasshoppers [25]. Over time, they learned that group life increases their chances of survival, and that they can have access to food sources more easily [26]. The life stages of a grasshopper and its life cycle as a creature with a group approach are shown in Fig. (4).

**Fig. 4:** The life stages of a grasshopper and its life cycle as a creature with a group approach.

The figure above shows that a cycle of grasshopper life includes its state of maturity, and at this stage of life, grasshoppers try to have access to optimal habitat and food situations through group and quasi-social behaviors. Lots of grasshoppers move and jump similar to spinning cylinders. In the following, by getting older, a group is made in the air by them. This indicates the way they migrate distant regions. The major attribute of the present sets within the larval step has been considered to be the slow motion and minor stages of the individuals [27]. Conversely, long and sudden motions have been considered to be a hallmark of the aforementioned groups amid more mature individuals. The discovery of resources of food has been regarded as an essential attribute of team life amid the individuals. Algorithms inspired by wildlife include two parts: exploitation and exploration. The candidates of search have been motivated to have unexpected motions in exploration, whereas they have a tendency of moving locally at operation time. The existing functions, also the looking for the objective, have been conducted unconsciously by the individuals. Studies show that a grasshopper can move under the problem space to be influenced through three elements: gravitational force, force of wind, and the force of motion towards the community and mass of grasshoppers. To model the grasshopper optimization algorithm, wind, gravity, and motions of the optimal solution can serve to alter the individuals' location. The model of mimicking the individuals' group manner has been formulated mathematically below[equation (9)]:

(9) $$X_{i}=r_{1}S_{i}+{r_{2}G}_{i}+r_{3}A_{i}$$

In this regard, $r_{1}$, $r_{2}$ and $r_{3}$ are three stochastic values in the range [0, 1], and $X_{i}$ specifies the location of the $i^{th}$ individual. $S_{i\;}$ denotes social interaction, $G_{i\;}$ refers to the gravitational force of the grasshopper i, and $A_{i\;}$ defines the wind's horizontal force. The subsequent formulas can be used for modelling the aforementioned vectors [equations (10), (11), (12)]:

(10) $$S_{i}=\sum_{j=1}^{N}=s\left(d_{ij}\right){\hat{d}}_{ij}$$

(11) $$G_{i}=-g.{\bar{e}}_{g}$$

(12) $$A_{i}=u.{\bar{e}}_{w}$$

In this relation, $d_{ij}$ defines the distance between the two grasshoppers i and j of the population of grasshopper, ${\hat{d}}_{ij\;}$ has been considered to be the element vector for displacement of individual, $s\left(d_{ij}\right)$ refers to a function to describe the social powers' influence, and $G_{i}$ specifies the gravitational force of the grasshopper i. In Eq. (11), the constant of gravity is ${\bar{e}}_{g}$ and illustartes a single vector towards the earth. The following equations illustartes the distance between two locusts single vectors to move the grasshopper and the its social force function as equations (13), (14), (15):

(13) $$d_{ij}=\left|X_{j}-X_{i}\right|$$

(14) $${\hat{d}}_{ij}=\frac{\left|X_{j}-X_{i}\right|}{d_{ij}}$$

(15) $$s\left(d_{ij}\right)=fe^{\frac{-r}{1}}-e^{r}$$

In the social force function, f illustrates the strength of gravity; moreover, r defines the proportion of the gravity dimension. By placing the values of $S_{i}$, $G_{i}$, and $A_{i}$ in the equation, the subsequent formula can be utilized [equation (16)]:

(16) $$X_{i}^{d}=c\left(\sum_{\begin{array}{c} j=1\\ j\neq i \end{array}}^{N}c\frac{{ub}_{d}-{lb}_{d}}{2}s\left(\left|X_{j}^{d}-X_{i}^{d}\right|\right)\frac{X_{j}-X_{i}}{d_{ij}}\right)+{\hat{T}}_{d}$$

where, ${ub}_{d}$ denote the higher limit, ${lb}_{d}$ define the minimum bound within the $D^{th}$ dimension, ${\hat{T}}_{d}$ has been considered to be the value of the $D^{th}$ dimension within the objective (the optimum solution ever achieved), and c has been regarded as the coefficient of decrease to diminish the gravity, comfort, and repulsion zone. Parameter c ought to decrease in proportion to the iterations' quantity. The present mechanism increases the amount of communications in operation. The coefficient c decreases the comfort zone according to the interactions' amount and is achieved in the following way [equation (17)]:

(17) $$C=c_{\max}-l\frac{c_{\max}-c_{\min}}{L}$$

where, $c_{\max}$ defines the highest amount, $c_{\min}$ denotes the lowest amount, l illustrates the present interaction; in addition, L refers to the highest quantity of interactions.

### 3.2 Amended Grasshopper Optimizer

The Amended Grasshopper Optimizer (AGO) is an enhanced iteration of the initial Grasshopper Optimizer algorithm. Although the original algorithm is effective and yields satisfactory outcomes for various problems, it does have certain limitations. These limitations include the tendency to become trapped in local optima and the occurrence of premature and improper convergence. In order to tackle these issues, this research proposes two modifications aimed at improving the algorithm's performance. The first modification involves incorporating chaos theory to enhance the stochastic values utilized within the algorithm. In the original Grasshopper Optimizer, the parameters $r_{1}$, $r_{2}$, and $r_{3}$ are random values that occasionally result in premature convergence [28,29]. To overcome this problem, the singer mapping mechanism is employed, which transforms these stochastic values into a more regular arrangement. The updated equations for determining the new values of $r_{1}$, $r_{2}$, and $r_{3}$ are as follows [equations (18), (19), (20)]:.

(18) $$r_{1}^{i+1}=1.07\left(7.9r_{1}^{i}-23.3{\left(r_{1}^{i}\right)}^{2}+28.7{\left(r_{1}^{i}\right)}^{3}-13.3{\left(r_{1}^{i}\right)}^{4}\right)$$

(19) $$r_{2}^{i+1}=1.07\left(7.9r_{2}^{i}-23.3{\left(r_{2}^{i}\right)}^{2}+28.7{\left(r_{2}^{i}\right)}^{3}-13.3{\left(r_{2}^{i}\right)}^{4}\right)$$

(20) $$r_{3}^{i+1}=1.07\left(7.9r_{3}^{i}-23.3{\left(r_{3}^{i}\right)}^{2}+28.7{\left(r_{3}^{i}\right)}^{3}-13.3{\left(r_{3}^{i}\right)}^{4}\right)$$

The Quasi-opposition learning procedure is the second modification implemented to address premature convergence. This technique involves comparing the newly generated population in the next iteration with their symmetric counterparts. The individual that performs better is chosen as the new candidate within the population. To determine the symmetric value of an individual, denoted as $X_{i}$, within the solution space bounded by Lb and Ub, equation (21)is utilized:

(21) $${\bar{X}}_{i}=Lb_{i}+Ub_{i}-X_{i}\;i=1,2,\ldots ,d\text{.}$$

The dimensionality of the problem is represented by the symbol d. Additionally, the equation below is used to calculate the Quasi-opposite value of $X_{i}$ [equation (22)].

(22) $${\overset{═}{X}}_{i}=rand\left(X_{i},0.5\times Lb_{i}+Ub_{i}\right)$$

where, ${\overset{═}{X}}_{i}$ defines the Quasi-opposite value of the $X_{i}$.

The Amended Grasshopper Optimization algorithm endeavors to enhance the overall performance of the original Grasshopper Optimizer by employing these modifications. Its objective is to address the issues of premature convergence and premature convergence, thereby improving its effectiveness in solving optimization problems.

### 3.3 Validation of algorithm

In order to validate the recommended Amended Grasshopper Optimization Algorithm (AGOA), the algorithm has been conducted on five cost functions, which were standard. The utilized test functions have been tabulated in Table 1.

**Table 1:** Utilized benchmark functions.

Function	Range	$f_{\min}$
$F_{1}\left(x\right)=\sum_{i=1}^{n}x_{i}^{2}$	[-100,100]	0
$F_{2}\left(X\right)=\sum_{i=1}^{n-1}\left[{\left(x_{i}+0.5\right)}^{2}\right]$	[-100,100]	0
$F_{3}\left(x\right)=\sum_{i=1}^{n}{|x}_{i}|+\prod_{i=1}^{n}\left|x\right|$	[-30,30]	0
$F_{4}\left(x\right)=\sum_{i=1}^{n}{ix}_{i}^{4}+random[0,1)$	[-128,128]	0
$F_{5}\left(x\right)=\sum_{i=1}^{n-1}\left[100{\left(x_{i+1}-x_{i}^{2}\right)}^{2}+{\left(x_{i}-1\right)}^{2}\right]$	[-128,128]	0

After validation of the Amended Grasshopper Optimizer on the five cost functions, the accomplishments have been compared to some modern techniques, such as the Locust Swarm (LS) optimization [20], Black Hole (BH) [30], Lion Optimization Algorithm (LOA) [31], Spotted Hyena Optimizer (SHO) [32], and the Basic Grasshopper Optimizer [33]. The parameter setting of all studied optimizers are stated below.

- LS (Locust Swarm) optimization [20]:

L=1;F=0.6;g=20

- Black Hole (BH) [30]:

a=0.5; Number of stars = 100

- Lion Optimization Algorithm (LOA) [31]:

This algorithm has some features which will be explained in the following. Prides' quantity = 5; nomad lions' percent = 30%; percent of roaming = 40%; probability of mutate = 0.1; rate of sex = 0.85; probability of mating = 0.4; and rate of Immigrate = 0.5.

- Spotted Hyena Optimizer (SHO) [32]:

$\vec{M}$ = 0.6; $\vec{h}$ = 5

- Grasshopper Optimization Algorithm (GOA) [33]:

c=0.01

For providing a fair and consistant outcomes, all of the algorithms are accomplished 35 times for each benchmark function, and their average value and STD value are provided for the validation. The population and the maximum value of all optimizers are considered to be 50 and 100, respectively. The optimizers are programmed by MATLAB R2017b environment. Table 2 illustrates the configuration of the system.

**Table 2:** Detail of the system.

Name	Setting
Hardware	Intel® Core™ i5-2410 M
CPU	2.3 GHz
RAM	8 GB
Frequency	2.3 GHz
Operating system	Windows 10
Programming software	MATLAB R2016b

Table 3 tabulates simulation achievements of the Amended Grasshopper Optimization Algorithm compared to several modern algorithms applied to the benchmark functions.

**Table 3:** Simulation accomplishments of the studied optimizers utilized in the cost functions.

Benchmark function	Metric	LS [20]	LOA [31]	SHO [32]	GOA [33]	AGOA
$F_{1}$	AVE	6.25 E−5	5.84 E−7	5.18 E−8	5.89 E−10	8.64 E−11
	STD	8.31E-5	7.93E-7	9.01E-9	3.25E-11	2.55E-12
$F_{2}$	AVE	45.54	35.93	27.98	13.16	1.0051
	STD	30.17	27.35	19.74	10.53	1.0001
$F_{3}$	AVE	2. 04	1. 92	1.13	0.84	0.01
	STD	1.84	1.52	1.01	0.14	0.041
$F_{4}$	AVE	1.05E-1	1.115	1.052	1.027	1.012
	STD	0.025	0.11	0.008	0.006	0.002
$F_{5}$	AVE	0.43	0.27	0.22	0.11	0.11
	STD	1.27E-3	3.71E-4	4.02E-5	6.18E-6	7.94E-7

Based on the table above, the suggested AGOA delivers the minimum AVE values for five studied cost functions that indicates its better precision in solving the analyzed functions towards some latest optimizers. Similarly, with analyzing the standard deviation values, it is observed that the proposed AGOA denotes the lowest quantity of the cost functions depicting the method's advanced reliability during different runs.

## 4 The optimized AlexNet/ELM network

The current part describes the approach of applying the suggested Amended Grasshopper Optimizer for providing an optimal configuration for the combined Alexnet and ELM network. The algorithm uses batch normalization technique during the optimization. For desingning the proposed network, the AlexNet is previously trained in the beginning. This pre-training is established to extract the dermoscopy images features. Afterward, batch normalization has been applied to determine the internal covariate shifting problem. Because the utilized network is a pre-trained network (with 1000 classes) and has a determined numbers of outputs, it should be adjusted and changed to a two-folded classifier, including healthy and tumor samples.

In this study, there are also six normalization layers which are placed after the pooling layer and the convolution layer. Afterward, the ELM network is placed at the classification layer of the network. In this manner, the number of layers have been achieved experimentally. To provide more efficient classification, the Amended Grasshopper Optimizer has been used to select the amount of the weights and the biases of the ELM net in the ALexNet. This is established by aiming to minimize the following target [equation (23)]:

(23) $$f\left(w,b\right)=\sum_{k=1}^{M}{\left(D_{k}-H_{k}\right)}^{2}$$

where, M signifies the quantity of training samples; additionally, $D_{k}$ and $H_{i}$, in turn, denote the intended value and the network's output.

The proposed method's architecture comprises three primary components: an AlexNet for extracting features, an ELM network for classification, and an AGOA for optimizing parameters. A summary of the network's architecture can be found in Table 4.

**Table 4:** Summary of the network's architecture.

Layer	Type	Input	Output	Activation	Batch normalization
1	Convolution	227x227x3	55x55x96	ReLU	Yes
2	Max pooling	55x55x96	27x27x96	–	–
3	Convolution	27x27x96	27x27x256	ReLU	Yes
4	Max pooling	27x27x256	13x13x256	–	–
5	Convolution	13x13x256	13x13x384	ReLU	Yes
6	Convolution	13x13x384	13x13x384	ReLU	Yes
7	Convolution	13x13x384	13x13x256	ReLU	Yes
8	Max pooling	13x13x256	6 × 6 × 256	–	–
9	ELM	9216	2	Linear	–

The network takes a brain MRI image of size 227×227×3 as input and generates a binary label to indicate the presence or absence of a tumor. To improve the training process and address the internal covariate shift problem, batch normalization layers are added after specific convolution layers (first, third, fifth, sixth, and seventh). This not only speeds up the training but also mitigates the internal covariate shift issue.

To simplify the network and avoid potential issues, like overfitting, local minima, and gradient vanishing, the fully connected layers of the original AlexNet are replaced with an ELM network. The ELM network is a single hidden layer feedforward network with random weights and biases.

To optimize the parameters of the ELM network, such as the number of hidden nodes, weights, and biases, the network utilizes the Amended Grasshopper Optimization Algorithm (AGOA). This algorithm enhances the accuracy and efficiency of the classification process.

During the training process, the network uses a learning rate of 0.01 and a batch size of 32; moreover, it performs 50 epochs. The convolution layers employ the ReLU activation function, while the ELM layer uses a linear activation function. For the output layer, the network applies a cross-entropy loss function and a softmax function.

## 5 Experimental results

The proposed method for the diagnosis of brain tumors has been implemented using image processing in MATLAB R2019b environment. Brain MRI images have been collected from “Brain-Tumor-Progression” [13], and they have been used to assess and contrast the efficacy of the suggested technique. For providing a proper assessment of the approach, it is analyzed based on some measurement indicators, including Matthew's Correlation Coefficient (MCC), F-score, accuracy, sensitivity, precision, and specificity. In the following, the explanation of all indicators has been given.

- Matthew's Correlation Coefficient (MCC):

This indicator considers true negative and positive as (TN) and (TP) and false negative and positive as (FN) and (FP) to assess even if the classes have different sizes. The MCC is a correlation coefficient between the predicted and the observed classifications. The MCC yields a value between −1 and 1. Where, 1 defines a faultless prediction, and −1 defines total disagreement between the predicted and the observed classification. The mathematical formula of this indicator is given below [equation (24)]:

(24) $$MCC=\frac{TN\times TP-TP\times FN}{\sqrt{\left(FP+TP\right)\times \left(FN+TP\right)\times \left(FP+TN\right)\times \left(FN+TN\right)}}\times 100$$

- Accuracy:

This illustrates the ratio of the accurately labeled tumors or healthy images to the total number of samples. Indeed, this indicator tells us how many images are correctly labeled out of all the samples. The existing indicator has been obtained via the subsequent formula [equation (25)]:

(25) $$Accuracy=\frac{TP+TN}{TP+TN+FP+FN}\times 100$$

- Sensitivity:

This indicator illustrates the proportion of the properly categorized tumors to the sum of samples that are really tumorous. This indicator tells us how many of all tumorous samples are correctly determined. The formula of the sensitivity has been calculated mathematically in the following way [equation (26)]:

(26) $$Sensitivity=\frac{TP}{TP+FN}\times 100$$

- Precision:

This indicator illustrates the propotion of the properly categorized tumors to the sum of samples that are labeled tumorous. This indicator tells us how many of them labeled as tumorous are really tumorous. This indicator is achieved by equation (27):

(27) $$Precision=\frac{TP}{TP+FP}\times 100$$

- Specificity:

This indicator determines the properly categorized healthy to the sum of samples that are indeed tumorous. This indicator tells us how many of the people that are tumorous, are labeled correctly. The specificity is formulated in the following way [equation (28)]:

(28) $$Specificity=\frac{TN}{TN+FP}\times 100$$

- F1-score:

This indicator includes both precision and sensitivity. The F1-score shows the mean value of the precision and sensitivity. This indicator provides the best results if there exists an appropriate balance between sensitivity and precision within the system. The present indicator has been formulated below equation (29):

(29) $$F1-score=2\times \frac{Precision\times Sensitivity}{Precision+Sensitivity}\times 100$$

The comparison results of the proposed method with some latest techniques, including AlexNet [34], CNN [35], and ELM [36], are stated within Table 5.

**Table 5:** Comparison achievements of the proposed technique with some latest techniques.

Technique	Accuracy	Precision	Specificity	F1-score	Sensitivity	MCC
ELM [36]	0.79	0.92	0.95	0.88	0.79	0.60
CNN [35]	0.95	0.93	0.93	0.90	0.88	0.88
AlexNet [34]	0.87	0.88	0.86	0.79	0.85	0.85
Proposed method	0.96	0.94	0.96	0.96	0.94	0.90

Fig. (5) present a graphical representation of the comparison achievements.

According to Table 5 and its illustration in Fig. (5), the proposed approach with 96 % accuracy can provide the maximum value toward the rest contrasted methods. Likewise, CNN-based method and AlexNet-based method with 95% and 87% are located in the 2nd rank and the 3rd rank, respectively. Finally, ELM-based method with 79% accuracy is located in the last rank. Furthermore, the proposed technique with 94% sensitivity is considered as the topmost amount toward the rest which shows its higher reliability in diagnostic task. The other indicators are also based on the explanations from Eqs. (24), (25), (26), (27), (28), (29), and the recommended approach denotes the best value for all of them.

**Fig. 5:** Comparison achievements of the technique method with some latest techniques.

For getting an additional investigation on the suggested technique, it also was put in comparison with several latest methods with completely different configurations, including Khan [37], Narmatha [38], Li [39], Mohammed [40], and Amin [41]. Here, two different indicators, including PPV (Positive Predictive Value) and NPV (Negative Predictive Value), and measures, like Sensitivity, Accuracy, and Specificity have been utilized. The mathematical formula of these indicators are given equations (30), (31):

(30) $$PPV=\frac{TP}{TP+FP}\times 100$$

(31) $$NPV=\frac{TN}{TN+FN}\times 100$$

Table 6 tabulates the comparison achievements of the proposed technique with some latest techniques.

**Table 6:** Comparison results of the proposed technique with some latest techniques.

Technique	Sensitivity	Specificity	PPV	NPV	Accuracy
Suggested technique	0.94	0.96	0.86	0.88	0.96
Khan's [37]	0.86	0.88	0.80	0.78	0.87
Narmatha's [38]	0.82	0.73	0.70	0.92	0.78
Li's [39]	0.71	0.69	0.66	0.85	0.76
Mohammed's [40]	0.79	0.69	0.67	0.88	0.73
Amin's [41]	0.77	0.85	0.75	0.79	0.80

Fig. (6) shows a graphical illustration of the results for more clarification.

Based on Table 6 and its illustration in Fig. (6), the recommended strategy with 96 % accuracy has still the finest value against Khan [37], Amin [41], Narmatha [38], Li [39], and Mohammed [40] with values of 87%, 80%, 78%, 76%, 73% that have been placed in the next ranks. Also, high NPV and PPV value for the suggested technique toward the other latest techniques illustrate the model's better occurrence condition for adjusting the likelihood of examination to recognize the tumor. Moreover, high value of the specificity of the recommended approach illustrates its higher occurrence-autonomous results.

**Fig. 6:** Comparison achievements of the proposed technique with some latest techniques.

## 6 Discussions

In this research paper, an efficient approach has been introduced for diagnosing brain tumors using a deep neural network that is based on metaheuristics. The approach combines an AlexNet for extracting features, an ELM network for classification, and an AGOA for optimizing parameters. To evaluate the effectiveness of the method, experiments have been conducted on a dataset consisting of 20 patients with newly diagnosed glioblastoma, and the results have been compared with other advanced techniques in the field.

The outcomes of the experiments demonstrated that the method outperformed the other techniques in terms of accuracy, precision, specificity, F1-score, sensitivity, and MCC, achieving values of 0.96, 0.94, 0.96, 0.96, 0.94, and 0.90, respectively. Furthermore, the robustness and stability of the method have been assessed by subjecting it to different levels of noise and image resolutions. In this section, we delve into the significance, implications, and meaning of our results, as well as the limitations and suggestions for future research. Findings strongly indicate that this method is highly effective in diagnosing brain tumors using MRI images. This is achieved by extracting intricate and high-level features from the images, reducing the complexity and computational burden of the network, and optimizing its parameters.

The approach demonstrated superior performance compared to existing methods that solely utilized CNNs or ELMs, as well as other metaheuristic algorithms like the chaotic bat algorithm or original grasshopper optimization algorithm. This indicates that this approach has the capability to accurately capture the subtle and unique features of brain tumors, enabling a fast and reliable diagnosis. Moreover, the approach contributes to the advancement of medical image analysis, particularly in the field of brain tumor diagnosis. It fills a gap in the existing literature by combining deep learning and metaheuristic techniques, which have been rarely explored together for this purpose.

Additionally, the method addresses a real-world problem as brain tumors are prevalent and highly lethal, emphasizing the importance of timely diagnosis for effective treatment and prognosis. By enhancing diagnostic accuracy and efficiency, it has the potential to assist clinicians and radiologists in reducing human errors and biases. However, it is important to acknowledge the limitations of this approach, which impact the validity and generalizability of the findings. Firstly, the evaluation was conducted on a relatively small and homogeneous dataset consisting of 20 patients with glioblastoma, a specific type of brain tumor. Therefore, the applicability of the method to other brain tumor types or different populations with varying characteristics, such as age, gender, ethnicity, or health status, may be limited.

Secondly, the effectiveness of the approach relies on the quality and availability of MRI images, which can vary depending on the imaging equipment, scanning protocol, and image processing techniques utilized.

Hence, this study might not yield satisfactory results when applied to low-quality or noisy images, as well as images with varying formats or resolutions. Additionally, the use of a linear activation function in our ELM network could restrict the network's ability to capture complex and nonlinear relationships between input and output variables.

## 7 Conclusions

Tumor in brain is abnormal gathering of cells. The brain is surrounded by skull that is very hard. Any growth in this limited space can cause problems. Benign or malignant are two types of Brain tumors. The intracranial pressure increases with growth in the non-cancerous or malignant tumor. Therefore, early diagnosis of the tumors are so significant in healing the tumor. Image processing is an efficient technique that can help the doctors improve the detection's accuracy. Within the current research, a novel optimized configuration of a modified AlexNet has been employed for effcacious recognition of the tumor in brain. The AlexNet has been modified based on using an Extreme Learning Machine (ELM) network in its classification layer. For optimizing the efficiency of the suggested technique, an Amended design of Grasshopper Optimizer has been designed and applied. This method considered biases and weights of the network as decision variables for achieving the lowest error amount between the desired and the model's output. The final accomplishments of the recommended strategy were compared to various modern techniques, and the simultions showed its higher efficiency for brain tumor diagnosis.

## Data availability statement

Research data are not shared.

## CRediT authorship contribution statement

**Jing Zhu:** Formal analysis, Data curation, Conceptualization. **Chuang Gu:** Formal analysis, Data curation, Conceptualization. **Li Wei:** Formal analysis, Data curation, Conceptualization. **Hanjuan Li:** Formal analysis, Data curation, Conceptualization. **Rui Jiang:** Formal analysis, Data curation, Conceptualization. **Fatima Rashid Sheykhahmad:** Formal analysis, Data curation, Conceptualization.

## Declaration of competing interest

The authors declare that they have no known competing financial interests or personal relationships that could have appeared to influence the work reported in this paper.
